This article has been retracted.

# Red Raspberry Extract Decreases Depression-Like Behavior in Rats by Modulating Neuroinflammation and Oxidative Stress

**DOI:** 10.1155/2022/9943598

**Published:** 2022-07-02

**Authors:** Yanhua Chen, Xia Yang, Hui Li, Jianqun Fang

**Affiliations:** ^1^Mental Health Center, General Hospital of Ningxia Medical University, Yinchuan, Ningxia 750001, China; ^2^Information Center, Health Commission of Ningxia Hui Autonomous Region, Yinchuan, Ningxia 750002, China; ^3^Minkang Hospital Department of Civil Affairs of Ningxia, Yinchuan, Ningxia 750011, China

## Abstract

**Objective:**

Red raspberry serves as a proven natural product to produce anti-inflammatory, antioxidant, and anticancer functions, but limited findings are available on its effects on depression. This study, by using a chronic unpredictable mild stress- (CUMS-) induced depression model, thus investigated the effects and underlying mechanism of red raspberry extract (RRE) on depressive behavior, inflammation, and oxidative stress.

**Methods:**

Different treatments were given after random grouping of Sprague-Dawley rats, including no intervention (control), CUMS induction, and CUMS+different concentrations of RRE, and subsequently, depression-like behavior tests were performed. HE staining was designed to observe the pathological damage of the hippocampal tissue in rats. The levels of oxidative stress, endocrine hormones, and inflammatory factors were determined by biochemical assay and ELISA, and gene expression (mRNA and protein) in the hippocampal tissue by qRT-PCR and Western blot.

**Results:**

On completion of CUMS treatment, the rats showed severe depression-like behavior, with obvious hippocampal tissue damage, oxidative inflammatory response, and endocrine imbalance. Importantly, RRE treatment significantly improved such depression-like behavior and attenuated histopathological damage in CUMS rats when reducing inflammation and oxidative stress and endocrine imbalance with upregulation of glutathione (GSH), superoxide dismutase (SOD), and interleukin- (IL-) 10 and downregulation of adrenocorticotropic hormone (ACTH), corticosterone (CORT), malondialdehyde (MDA), IL-1*β*, cyclooxygenase- (COX-) 2, and human macrophage chemoattractant protein- (MCP-) 1. In addition, for CUMS rats, RRE was a contributor to increasingly expressed brain-derived neurotrophic factor (BDNF), neurotrophic tyrosine receptor kinase 2 (TrkB), and p-mTOR but inhibited p-GSK-3*β* expression in the hippocampal tissue. All the above antidepressant effects of RRE were concentration-dependent.

**Conclusion:**

By regulating neuroinflammation, oxidative stress response, endocrine level, and BDNF/TrkB level, RRE showed potential efficacy in alleviating depression-like behavior and histopathological damage of hippocampal tissue in CUMS rats by regulating the GSK3*β* and mTOR signaling pathways.

## 1. Introduction

Depression, the second most disabling condition worldwide, is a mental disorder that causes serious harm to human health. It is characterized by persistent low mood, slow thinking, anhedonia, disturbed sleep, and appetite loss. In severe cases, the patients may self-mutilate and commit suicide [1, 2]. Epidemiological surveys have found an increase in the year by year incidence, disability, and mortality of depression in recent years [3]. Moreover, depression has severe impacts on a person's physical and mental health and social economy, accounting for 10.3% of the total disease burden [4, 5]. Depression is a multifactorial disease attributed to heredity, environment, epigenetics, and others, whose underlying mechanism is complex and has not yet been elucidated [6], thereby making its clinical diagnosis and treatment difficult. Meanwhile, most antidepressant drugs are associated with severe adverse events and unsatisfactory responses. Therefore, finding new and effective drugs with fewer side effects for treating depression is important.

Red raspberry (Rubus idaeus L. (RB)) is a berry of the Rosaceae family. It contains various essential nutrients and active compounds, such as anthocyanins, tannin, brass, organic acids (including phenolic acids), fatty acids, xylan, and superoxide dismutase (SOD) [7, 8], which have been shown to have antioxidant, anti-inflammatory, and anticancer functions and other pharmacological effects [9, 10]. RB can inhibit the production of superoxide anion in the heart and aorta of obese mice and promote the activities of hepatic glutathione peroxidase and superoxide dismutase [11]. Also in obese mice (liver tissue), NLRP3 inflammasome activation and production of interleukin- (IL-) 1*β* and IL-18 are shown to be inhibited as a consequence of RB treatment [12]. It has been reported that red raspberry extract (RRE) has a central role in several diseases, such as arthritis, whereby RRE can significantly inhibit inflammation and the onset of clinical symptoms [13, 14]. RRE, based on in vitro experiments by Zhang et al., suppresses hepatoma cell growth (HepG2 and Huh7 cells) through the PTEN/AKT signaling pathway [15]. However, the role of RRE in depression, however, is still unknown to the medical community.

In this study, for determining the effect and mechanism of RRE on depression, we traced the changes in depressive-live behavior, serum neuroendocrine hormone, inflammatory factors, and brain-derived neurotrophic factors in chronic unpredictable mild stress- (CUMS-) treated rats. The theoretical basis for the clinical treatment of depression can be derived from the research.

## 2. Materials and Methods

### 2.1. Model Establishment and Grouping

A CUMS-induced depression rat model was established as previously described [11]. Rats from the control group remained untreated, while the others were subjected to CUMS and randomly given two or three kinds of stimulation every day. The stimuli comprised of (a) moist bedding, (b) no water overnight, (c) overnight fasting, (d) tilting their cage to 45° for 24 h, (e) overnight light flashing, (f) reversal of day/night light cycle, (g) odor, (h) white noise at 80 dB for 3 h, (i) overnight staying in a crowded cage, (j) cold swimming at 8°C lasting 5 min, and (k) restraint behavior for 4 h. The same stimulation was given discontinuously for 4 weeks.

Fifty male Sprague-Dawley rats were acquired from the Shanghai Southern Model Organisms Center (Shanghai, China). These 6–8-week-old rats weighing 180–220 g were subjected to random grouping (*n* = 10, each group) which consisted of the control group, CUMS group, and three RRE groups (30 mg/kg, 60 mg/kg, and 120 mg/kg). Rats as controls were fed normally and given normal saline by gavage in the 3rd to 4th week. The remaining animals were also given gavage with normal saline or 30 mg/kg, 60 mg/kg, or 120 mg/kg RRE in the 3rd to 4th week, respectively, based on CUMS induction for 4 consecutive weeks (Figure 1). After completing the behavioral test, the rats in each group were sacrificed, followed by collection of their blood and brain hippocampal tissue for the next steps. This study was approved by the Ethics Committee of the General Hospital of Ningxia Medical University (Ningxia, China) (KYLL-2021-1080) and performed in accordance with the approval guidelines.

### 2.2. Behavioral Testing

#### 2.2.1. Weight Determination

The rats in each group were weighed every week, and the following formula was applied to the calculation of the change in body weight:

(1) $$\begin{array}{c} \text{Body weight change }\left(\%\right)=\frac{Wn-W0}{W0}\times 100\%. \end{array}$$

Here, *Wn* refers to the body weight on the last day of the *n*th week and W0 refers to the body weight on the last day of adaptive feeding.

#### 2.2.2. Sucrose Preference Test

The sucrose preference test (SPT) was performed as a measurement to evaluate the responsiveness of the rats to positive stimuli, including habituation training and formal testing. Sucrose AR grade reagent was purchased from Shanghai Sinopharm Co., Ltd. During the adaptation training, a bottle of 1% (*w*/*v*) sucrose solution (200 mL) and a bottle of pure water (200 mL) were placed in the rats' cage in sequence, and the order of the left and right liquids was switched after 12 h to prevent the rats from habitually drinking only one side of the liquid. Baseline measurements were recorded. During the formal test, the rats were fasted for 12 h and kept in separate cages with free access to sucrose solution (200 mL) and pure water (200 mL). After 12 h, the drinking consumption was recorded, and the water intake was measured once before and once after treatments. The following formula was applied to the quantization of sucrose preference [16]:

(2) $$\begin{array}{c} \text{Sucrose preference }\left(\%\right)=\frac{\text{sucrose solution intake}}{\text{water intake}+\text{sucrose solution intake}}\times 100\%. \end{array}$$

#### 2.2.3. Open Field Test

The open field test (OFT), a test to assess exploratory activity and anxiety-like behavior in open boxes, was performed using a square box (150 cm × 150 cm × 50 cm) as an open field. After being carefully placed in the center of the field without restriction of movement for 5 min, with traces of their movement by a video camera above them, SMART software served to analyze the total moving distance moved and time spent in the central area. The apparatus was wiped utilizing a damp cloth and then dried with a hot air blower after each test [17].

#### 2.2.4. Elevated Plus Maze

The elevated plus maze (EPM) is a common measure apparatus (100 cm above the floor) with two open arms and two closed arms, both measuring 50 cm × 10 cm × 40 cm. All the rats were transferred to the behavior testing room 15 min prior to the first trial for them to adapt to the environment, with the room volume maintained at 30 decibels as far as possible. After being gently placed in the center of the apparatus facing the open arms, the rats had no restriction of movement for a period of 5 min. Then, with records of their movement by a video camera above them, the calculation of open arm entries and time spent in open arms was achieved [18].

### 2.3. Forced Swim Test

The forced swim test (FST), an examination of depression-like behaviors, can be divided into a training and a testing phase [19]. The experiments were performed following the protocol of Rogoz et al. [20]. During the training phase, the rats were gently placed in a transparent cylindrical glass container with a water depth of 30 cm (50 cm in height and 23 cm in diameter) to swim alone for 15 min (water temperature 24°C ± 1°C). After 24 h, they were put into the water for the swimming test for 6 min. All test procedures were recorded from the other side of the cylinder by a camera. Their immobility time and swimming time were recorded.

### 2.4. Hematoxylin and Eosin (HE) Staining

On completion of drying at ambient temperature, the rats' hippocampal tissue sections were processed as follows: 30 s fixation (ambient temperature, 30 s), 2 s rinsing in 1x PBS, 60 s staining in hematoxylin (60°C), 10 s rinsing in 1x PBS, 3 s differentiation with 1% hydrochloric acid alcohol, 2 s rinsing in 1x PBS, 3 min staining in eosin, and 2 s rinsing in 1x PBS again. The treated sections were dehydrated using 70%, 80%, 95%, and absolute ethanol for a period of 5 min and washed using xylene (3 × 5 min). Finally, they were mounted by transparent neutral gum, followed by use of a microscope (BX63, Olympus, Japan) for observation and photograph.

### 2.5. Biochemical Tests

Saline was added to the rats' hippocampal tissues, which were then grounded into tissue homogenates using a tissue grinder. On completion of centrifugation, the supernatant was collected to dilute separately into different concentration gradients of stock solutions. Measuring the levels of malondialdehyde (MDA), superoxide dismutase (SOD), and glutathione (GSH) was achieved using an automatic biochemical analyzer following the instructions of the biochemical detection kit (Elabscience, China).

### 2.6. Enzyme-Linked Immunosorbent Assay (ELISA)

Adrenocorticotropic hormone (ACTH) and corticosterone (CORT) in serum and IL-1*β*, IL-10, cyclooxygenase- (COX-) 2, and human macrophage chemoattractant protein- (MCP-) 1 in the hippocampal tissues were measured on the basis of the instructions of the ELISA kit (Nanjing Jiancheng Bioengineering Institute, China). Homogenates of the hippocampal tissues were taken from the rats, and the supernatant was diluted, to which the sample/standard and reagents were sequentially added to the ELISA plate for the reaction. The absorbance (OD value) at 450 nm wavelength was detected using an ELISA plate reader. The levels of CORT, ACTH, IL-1*β*, IL-10, COX-2, and MCP-1 in the samples were calculated using the standard curve.

### 2.7. Real-Time Quantitative Reverse Transcription PCR (qRT-PCR)

Determination of the concentration of total RNA was carried out with the Nanodrop machine and total RNA extraction gained from hippocampal tissues using the Trizol reagent (Sigma, USA). Then, reverse transcription of RNA into cDNA was completed according to the reverse transcription kit instructions (Takara, Japan). The mRNA expression level was detected following the instructions of the fluorescence quantitative kit (Takara, Japan). The 2^−*ΔΔ*Ct^ method was used for data analysis [21], and GAPDH served to provide an internal reference. The primer sequences used are displayed in Table 1.

### 2.8. Western Blot

Determination of the concentration of total protein was carried out with a BCA kit and with total protein extraction gained from hippocampal tissues using the Trizol reagent (Beyotime, China). Then, after separation using SDS-PAGE, the protein was blotted onto the polyvinylidene fluoride (PVDF) membrane by wet transfer. Next, total protein was then blocked using 5% nonfat dry milk for 2 h and subsequently incubated overnight at 4°C with the primary antibodies (BDNF, TrkB, mTOR, p-mTOR, GSK-3*β*, p-GSK-3*β*, and *β*-actin). On the following day, the rinsing step using phosphate buffer was carried out first, and subsequently, the membrane was subjected to 1 h of incubation with secondary antibodies at ambient temperature. Then, ECL was added after thorough washing, and the FliorchemHD2 imaging system was used for scanning and analysis [22]. Quantification of immunoreactive bands was conducted using ImageJ software, with *β*-actin as the internal reference.

### 2.9. Statistics

The data were analyzed using SPSS 21.0 employed for analyzing data, with statistics in the form of the mean ± standard deviation (SD). Comparison between two groups and multiple groups was made using a *t*-test and one-way analysis of variance, respectively. *P* < 0.05 served as the criterion to determine the significance of difference.

## 3. Results

### 3.1. RRE Significantly Inhibits Depression-Like Behavior in CUMS Rats and Ameliorates Histopathological Damage in the Hippocampal Tissue

We first used the CUMS method to establish a rat model for depression. Before the experiments, the initial body weight of the rats in each group had no marked difference. To determine the effects of CUMS and RRE on depression-like or anxiety behaviors in rats, we evaluated the behaviors of the rats in each group via SPT, OFT, and FST. Comparison between the control and CUMS groups and between the CUMS and RRE groups revealed that CUMS cause significant weight change in the rats over four weeks, but the change could be restored after RRE treatment (Figures 2(a) and 2(b)). Further, CUMS treatment was associated with a reduction in sucrose preference and worse performance in OFT (decreases in time spent in the central area and total movement distance), EPM (decreases in time spent in open arm and open arm entries), and FST (decreased swimming time and prolonged immobility time). The above depression-like behaviors were significantly improved by gavage of RRE in a concentration-dependent manner (Figures 2(c)–2(i)).

The pathological changes of hippocampal tissues were further assessed by HE staining. We found obvious pathological damage to hippocampal tissue in the CUMS group, which could be alleviated to different degrees by RRE treatment (Figure 2(j)). The above results showed that we had successfully established a CUMS-induced depression model and that RRE treatment could significantly inhibit depression-like behavior and improve the histopathological damage of the hippocampal tissue in CUMS rats.

### 3.2. RRE Decreases the Levels of ACTH and CORT in the Serum of CUMS Rats

ACTH and CORT, as previously reported, have higher levels in patients with depression [23]. We also confirmed CUMS induced increased serum levels of ACTH, and CORT in the serum of rats in the CUMS was markedly increased but could be reduced by RRE in a concentration-dependent manner (Figures 3(a) and 3(b)).

### 3.3. RRE Reduces Inflammatory Responses in Hippocampal Tissue of CUMS Rats

Depression development has an association with inflammatory cytokines secreted by the activated immune system [24]. We measured the levels of proinflammatory factors (IL-1*β*, COX-2, and MCP-1) and anti-inflammatory factor IL-10 in the hippocampal tissue in each group using ELISA to look into what effect RRE had on neuroinflammation in CUMS-treated rats. In comparison with the control group, the CUMS group presented with a significant elevation of IL-1*β*, COX-2, and MCP-1 expression in the hippocampal tissue (Figures 4(a)–4(d)), while IL-10 expression had a marked reduction. Further, a dose-dependent decline in the levels of IL-1*β*, COX-2, and MCP-1 and an increase in IL-10 occurred as a consequence of RRE treatment.

### 3.4. RRE Inhibits Oxidative Stress Response in Hippocampal Tissue of CUMS Rats

To explore the effect of RRE on the oxidative stress response of CUMS rats in each group, we examined the content of oxidative stress-related molecules in the hippocampal tissue of rats using biochemical tests. The CUMS rats had relatively high levels of GSH and SOD and low levels of MDA, but administration of RRE increased the GSH and SOD levels and decreased the MDA level in a dose-dependent manner (Figures 5(a)–5(c)).

### 3.5. RRE Promotes the Expression of BDNF and TrkB in the Hippocampal Tissue of CUMS Rats

In this study, qRT-PCR and Western blot were conducted to detect the expression of BDNF and TrkB in the hippocampal tissues of rats in each group. The results in the hippocampal tissue showed decreased protein and mRNA expression levels of TrkB and BDNF after CUMS treatment (Figures 6(a)–6(c)). However, after administration of RRE treatment in different concentrations, the two were increased significantly, except for the mRNA expression levels of TrkB in CUMS rats in the RRE 30 mg/kg group which remained almost unchanged.

### 3.6. RRE Regulates mTOR and GSK-3*β* Signaling in the Hippocampal Tissue of CUMS Rats

As reported, the mTOR pathway was involved in depression and antidepression [25], and the GSK-3*β* pathway was shown to regulate learning and memory impairment in depressed rats [26]. Here, we attempted to give an account of the possible mechanism of RRE in CUMS rats by detecting relevant protein levels of the mTOR and GSK-3*β* signaling pathways. As shown in Figures 7(a) and 7(b), the phosphorylation level of mTOR and the ratio of p-mTOR/mTOR in the hippocampal tissue presented with reduction in CUMS rats compared with those receiving no interventions, while the phosphorylation level of GSK-3*β* was significantly increased and the ratio of p-GSK-3*β*/GSK-3*β* significantly increased. RRE treatment could reverse the changes in the expression of the above proteins.

## 4. Discussion

Globally, the CUMS model is one of the classic depression models widely recognized by researchers [27] for searching for depression, a psychiatric disorder with high prevalence [6]. According to our experiments, a decline was identified in CUMS rats in body weight, preference for sucrose, time spent in the central area and total distance traveled in OFT, time spent in open arms and open arm entries in EPM, and swimming time in FST. Moreover, as confirmed by HE staining, the hippocampal tissue of CUMS rats displayed obvious pathological damage, which indicated the successful establishment of the depression model. In addition, administration of different concentrations of RRE significantly improved the body weight change, sucrose preference, free movement ability, memory, and pathological damage of rats to varying degrees. This evidence indicates that RRE is a contributor to alleviating depression-like behaviors like anhedonia, bradykinesia, and histopathological damage in the hippocampal tissue of CUMS rats by having an antidepressant effect that was directly proportional to its concentration.

Studies have found that the abnormal excitation of the hypothalamic-pituitary-adrenal axis is closely related to depression. Stress may promote the release of serum CORT, corticotropin-releasing hormone, and ACTH in rats by inducing the activation of the HPA axis to deregulate its negative feedback regulation, damaging tissues such as the hippocampus and prefrontal cortex, and further leading to depression and cognitive impairment [28]. In this study, observation of CORT and ACTH in serum produced an increased result in CUMS rats, and RRE treatment could significantly inhibit the increase in ACTH and CORTs.

Patients with depression are usually associated with increased secretion of cytokine IL-1*β* and decreased IL-10 and a significant increase in the expressions of proinflammatory genes COX-2 and MCP-1 [29–31]. Consistently, our work demonstrated that CUMS rat hippocampal tissue had greatly increased IL-1*β*, COX-2, and MCP-1, while IL-10 was significantly decreased. These changes, however, were reversed with the addition of RRE, indicating that regulation of the release of inflammatory factors could be the reason for RRE-caused relief of depression.

In recent years, investigators have explored whether an oxidative stress injury has a role as being a trigger for depression and what its mechanism is. In a physiological state, free radicals are normal metabolites in the process of mitochondrial circulation and oxidative phosphorylation, which can be eliminated by the body's SOD, GSH-PX, CAT, and other enzymes or nonenzymatic molecules such as vitamin C, vitamin E, and other antioxidant stress systems. In a pathological state, oxidative stress is dominant, and insufficiency in antioxidative stress function could lead to oxidative stress damage in the body. MDA, the main product of lipid peroxidation, has been used to reflect the degree of lipid peroxidative damage in the body [32]. The present study also found that the activities of GSH and SOD in CUMS rat hippocampal tissue significantly downregulated while upregulation occurred in the content of MDA, suggesting that the imbalance of oxidative stress in the brain may lead to peroxidative damage to neurons. The advent of RRE greatly restored the activities of GSH, and SOD were restored with the advent of RRE, accompanied by decreased MDA contents. The antioxidant effect of REE on CUMS rats was closely related to its concentration.

Besides, our study also found markedly decreased BDNF and TrkB in the hippocampal tissue from CUMS rats, but their expression could be greatly restored after RRE treatment. BDNF, known as brain-derived neurotrophic factor, is ubiquitous in the central nervous system and crucial to nervous system development and neuronal remodeling [33]. A significant decrease in BDNF expression has been noticed in the central nervous system and peripheral blood of patients with depression [34]. BDNF activates the intracellular functional region and triggers the autophosphorylation of TrkB by specifically binding to TrkB elements, thereby activating the downstream Ras-MAPK pathway to mediate synaptic plasticity and the growth and proliferation of hippocampal neurons. These processes may thereby maintain and promote memory and spatial recognition functions [35, 36]. The above studies suggest that the antidepressant effects of RRE on rats could be related to the reversal of the expression of BDNF and TrkB.

GSK-3 is a glycogen synthase kinase with two isoforms, *α* and *β*. GSK-3*β* is widely expressed in all brain regions [37]. Studies have shown that the phosphorylation level of GSK-3*β* is increased in depressed animals after stress. Injection of GSK-3*β*-specific inhibitor increased the content of *β*-catenin in the hippocampal tissue and rapidly produced an antidepressant effect [38]. The activity of brain tissue GSK-3*β* significantly increased in depression and suicidal patients [39]. mTOR is a serine/threonine kinase. Activation of mTOR could promote the synthesis of local synaptic proteins and the maturation and formation of new synapses, thereby affecting the pathogenesis of depression and antidepressant treatment. The mTOR signaling pathway has an impact on the efficacy of many classic antidepressants [40]. In this present study, CUMS rats showed decreased p-mTOR and reduced ratio of p-mTOR/mTOR in the hippocampal tissue, while phosphorylation of GSK-3*β* and the ratio of p-GSK-3*β*/GSK-3*β* greatly increased. In addition, RRE treatment activated the activity of mTOR and inhibited the activity of GSK-3*β*, suggesting that the protective effect of RRE on rat behavior could be related to the regulation of GSK-3*β* and mTOR signaling pathways, but the specific mechanism needs further experimental exploration.

Moreover, RRE contains a variety of active substances, such as tannin and anthocyanins. In this study, RRE was used to directly study the therapeutic effect, but its main components were not detected, and the separation and purification were not performed. Therefore, the specific active substances in RRE that exert antidepressant effects could not be determined, and the clarification of its active substances requires further isolation and experimental exploration. Nevertheless, there is no doubt that this study has depicted the important role of RRE in antidepressant therapy.

## 5. Conclusion

In summary, this study showed that RRE was associated with an improvement in CUMS-induced depression-like behavior and regulated inflammatory factor secretion, oxidative stress substance secretion, hormone levels, and the expression levels of BDNF and TrkB in CUMS rats. The antidepressant effects of RRE were related to the GSK-3*β* and mTOR signaling pathway. Although these could suggest a possible association between RRE and alleviation of hippocampal tissue damage, additional investigations are warranted to confirm these findings and shed more light on the possible underlying mechanism.

## Figures and Tables

**Figure 1:** Grouping treatment of Sprague-Dawley rats and the behavioral experimental process. W0-W4 represent the rat's body weight on the 0th to 4th week, respectively. OFT: open field test; FST: forced swim test; EPM: elevated maze test; SPT: sucrose preference test.

**Figure 2:** Effect of RRE on depression-like behavior and histopathological damage in the hippocampal tissues of rats in each group: (a, b) body weight of rats during weeks 0-4; (c) sucrose preference test before and after CUMS; (d, e) total distance moved; (d) time spent in the central area of rats (e) in open field test; (f, g) open arm entries (f) and time spent in open arms (g) in elevated plus maze test; (h, i) immobility (h) and swimming (i) time in force swim test; (j) HE staining showing the pathological damage of the hippocampal tissue. ^∗∗^*P* < 0.01*vs.* control group, ^##^*P* < 0.01*vs*. CUMS group.

**Figure 3:** Effects of RRE on ACTH and CORT levels in the serum of CUMS rats. (a, b) ELISA detecting the levels of CORT (a) and ACTH (b) in the serum: ^∗∗^*P* < 0.01*vs.* control group, ^##^*P* < 0.01*vs*. CUMS group.

**Figure 4:** Effects of RRE on neuroinflammation in CUMS rats. (a–d) The secretion levels of IL-1*β* (a), IL-10 (b), COX-2 (c), and MCP-1 (d) in hippocampal tissue measured by ELISA, ^∗∗^*P* < 0.01*vs.* control group, ^##^*P* < 0.01*vs*. CUMS group.

**Figure 5:** Effects of RRE on oxidative stress response in CUMS rats: (a–c) the contents of GSH (a), SOD (b), and MDA (c) in the hippocampal tissue determined by biochemical tests, ^∗∗^*P* < 0.01*vs*. control group, ^##^*P* < 0.01*vs.* CUMS group.

**Figure 6:** Effects of RRE on BDNF and TrkB expression levels in the hippocampal tissue of CUMS rats: (a) qRT-PCR was used to detect BDNF (a) and TrkB (b) expression in the hippocampal tissues; (c) Western blot to measure protein expression of BDNF and TrkB in the rats' hippocampal tissue. ^∗∗^*P* < 0.01 vs. control group, ^#^*P* < 0.05 and ^##^*P* < 0.01*vs*. CUMS group.

**Figure 7:** Effects of RRE on GSK-3*β* and mTOR signaling pathways in CUMS rats: (a) mTOR, p-mTOR, GSK-3*β*, and p-GSK-3*β* in the hippocampal tissue measured by Western blot; (b) grayscale analysis of p-mTOR/mTOR and p-GSK-3*β*/GSK-3*β* ratios. ^∗∗^*P* < 0.01 vs. control group, ^##^*P* < 0.01 vs. CUMS group.

**Table 1:** qRT-PCR primer sequences.

Gene names	Primer sequences (5′ to 3′)
BDNF	F AAAACCATAAGGACGCGGACTT
	R AAAGAGCAGAGGAGGCTCCAA
TrkB	F CACACACAGGGCTCCTTA
	R AGTGGTGGTCTGAGGTTGG
GAPDH	F AGTGCCAGCCTCGTCTCATA
	R GGTAACCAGGCGTCCGATAC

## Data Availability

The data used to support the findings of this study are available from the corresponding author upon request.
